The article "The Effect of Skin-to-Skin Contact on Postoperative Depression and Physical Recovery of Parturients after Cesarean Section in Obstetrics and Gynecology Department" was retracted in 2023. Reasons: signs of a paper mill; suspected computer-generated content; unreliable results or conclusions; concerns about the data.

# The Effect of Skin-to-Skin Contact on Postoperative Depression and Physical Recovery of Parturients after Cesarean Section in Obstetrics and Gynecology Department

**DOI:** 10.1155/2022/9927805

**Published:** 2022-01-22

**Authors:** Ying Zheng, Yanping Xia, Weijuan Ye, Congxia Zheng

**Affiliations:** ^1^Operating Room, The Maternity & Children Care Hospital of Lishui City, Lishui, Zhejiang, 323000, China; ^2^Gynecological Ward, The Maternity & Children Care Hospital of Lishui City, Lishui, Zhejiang, 323000, China; ^3^Nursing Department, The Maternity & Children Care Hospital of Lishui City, Lishui, Zhejiang, 323000, China

## Abstract

The effect of skin-to-skin contact (SSC) on postpartum depression and physical rehabilitation of cesarean section women was explored. 280 parturients undergoing cesarean section were selected and were rolled into two groups randomly. The parturients in the control group (Con group, 140 cases) received routine care, and those in the experimental group (Exp group, 140 cases) received SSC on the basis of routine care. The postpartum depression and physical recovery of parturients in two groups were compared. It was found that, in the Exp group, the number of pregnant women with no or with very mild depression was much more 85% vs. 55%), the number of women with adequate lactation was more (53 cases vs. 27 cases), the first lactation time (FLT) was dramatically shorter (41.25 ± 4.81 h vs. 58.43 ± 5.43 h), the breastfeeding success rate (BFSR) and breastfeeding rate (BFR) were obvious higher, the days for uterine involution was much shorter (6.96 ± 1.13 days vs. 9.47 ± 1.75 days), the descent of uterine fundus 24 hours after delivery (24 h-DUF) was obviously larger (3.17 ± 0.26 mm vs. 1.56 ± 0.43 mm), the duration of lochia (DOL) was remarkably shorter (33.21 ± 5.32 days vs. 25.32 ± 3.54 days), and the *Visual Analogue Scale* (VAS) score was lower (4.88 ± 0.32 points vs. 3.41 ± 0.53 points), showing statistical differences for all above indicators (*P* < 0.05). It suggested that SSC could effectively relieve the postpartum depression of uterine parturients, promote the lactation, increase the BFR, facilitate uterine involution, and alleviate chronic uterine inflammation and postpartum pain, showing high clinical application and promotion value.

## 1. Introduction

With the rapid development of the global economy, the proportion of women in the workplace is increasing, which also causes a lot of pressure on women from various aspects [1]. In many large cities, the rate of cesarean section is increasing year by year with the gradual increase in the number of elderly parturients and the increase in huge children [2]. Studies have shown that in the early 1990s, the cesarean section rate of urban women in China was not particularly high (15% ~20%), but it had soared to about 40% in 2003 [3]. Such a high rate makes it difficult for women to give birth to the second time, and the risks associated with them also increase [4]. Moreover, cesarean section will bring many complications to parturients after operation, such as postpartum hemorrhage, insufficient uterine contractility, wound infection, endometritis, urinary system infection, bladder or intestinal injury caused by surgery, postpartum pain, pelvic vein thrombosis, intraoperative bleeding, and many recent complications [5]. In addition, there will be complications such as uterine scar pregnancy, abnormal placenta position, and chronic pelvic inflammatory disease [6]. More importantly, the recovery of cesarean section parturients is not so fast compared to normal parturients, which is mainly reflected in breast secretion and wound pain. One of the obvious symptoms is postpartum depression in the parturient. There are many reasons for the occurrence of postpartum depression, such as the inability of parturients to quickly integrate into the mother's identity, the occurrence of a major event that causes a heavy psychological burden on the parturients, endocrine disorders, family history of depression, and physical diseases. And postpartum depression is also closely related to breastfeeding. Therefore, it is very necessary to find care methods that effectively help cesarean section parturients physical and psychological rehabilitation [7, 8].

Skin-to-skin contact (SSC) can also be called Kangaroo Mother Care (KMC), which mainly refers to a series of care methods such as premature infants who have skin contact with parturients at birth and breastfeeding [9]. Because of its simple operation, softness, and high efficiency, it is widely used in the care of newborns [10]. Many clinical experiments have proved that SSC can make the relationship between mother and child closer, which is conducive to the recovery of newborn's body temperature, accelerates metabolism, and maintains breathing [11]. Campbell-Yeo et al. (2019) [12] performed SSC on 50 preterm infants and compared with traditional care preterm infants; it was found that the body temperature recovery of the two groups of preterm infants was not much different, and their subsequent development indicators showed that SSC preterm infants had more advantages. Mazumder et al. (2019) [13] found that SSC not only stabilizes the basic physical indicators of premature infants but also improves cognitive function to a certain extent. It can be concluded from the previous studies that most of the current research on skin contact care is mainly focused on the recovery of newborns, but there are very few studies on the impact of the recovery of women born under cesarean section [14]. Based on this, 280 pairs of parturients and newborns that underwent cesarean section were selected and randomly rolled into two groups. The control group received routine care, and the experimental group received skin contact care on the basis of routine care. Postpartum depression, lactation, breastfeeding, uterine involution, lochia duration, and VAS pain score were compared between the two groups. It was hoped to provide clinical research data for the application of SSC in relieving cesarean section parturients postpartum depression and restoring physical health.

## 2. Objects and Methods

### 2.1. Research Objects

280 cesarean section parturients in the our hospital from February 18, 2019 to January 27, 2020 were included as the objects, and they were aged 20 to 38 years old. All objects were randomly rolled into two groups, and they received routine care in the control group (Con group, 140 cases) and SSC based on routine care in the experimental group (Exp group, 140 cases). The study had been approved by the Medical Ethics Committee of our hospital, and the parturients and their family members had learned about the study and signed the informed consent forms.

### 2.2. Inclusion Criteria

Women who met below requirements could be included: parturients of cesarean section delivery, parturients whose newborns showed Apgar scores of 8 ~ 10 points at 1 minute and 5 minutes, parturients with normal mental state, and parturients with signed informed consent.

### 2.3. Exclusion Criteria

Objects meeting below requirements had to be excluded: parturients who were unwilling to breastfeeding; parturients with symptoms such as diabetes and hypertension during pregnancy; parturients with infectious diseases, such as hepatitis B and syphilis; and parturients whose newborn needed to be rescued, leading to the separation of mother and child.

### 2.4. Care Methods

The routine care was performed for parturients in the Con group, and the specific operations were as follows. Firstly, the nurse cleaned the newborn's respiratory tract, cut the umbilical cord, and wiped off the blood on the newborn's body. After that, the length and weight of the newborn were measured and marked on the hand ring, the footprint of the newborn was recorded, and the vitamin K1 was injected. Thirdly, the newborn had to be treated with vaccinate and disease screen, and the diaper was worn. Fourthly, medical staff had to perform breast massage, perineum care, and psychological care on parturients and instruct parturients to hold the baby to promote breastfeeding proficiency. Fifthly, medical staff had to patiently answer the questions and solve the problems encountered by parturients and observe the vital signs of parturients and newborns at any time.

Parturients and newborns in the Exp group accepted SSC on the basis of routine care. The specific operations were as follows. Firstly, the family members were required to assist the parturients to remove the coat, expose the chest and abdomen, maintain a semirecumbent posture, and adjust the angle of the bed head to make the parturients comfortable. The newborn was allowed to be naked, lying prone between the breasts of the parturients, and keep head parallel to the breasts and slightly offset to one side, so as to maximize the contact area between the newborn and the parturients. Thirdly, the back and body of newborn were covered with a blanket, while parturient was required to hold the newborn's buttocks with one hand and to embrace the newborn's back with the other hand to prevent the newborn from slipping. Then, the parturients and the newborn should be given continuous SSC within three days of hospitalization, with twice a day. The newborn should be given SSC for one hour after the bath in the early morning and at 4 : 00~5 : 00 pm. After being discharged from the hospital, the medical staff had to tell parturients to perform SSC by phone for about one month.

### 2.5. Observation Indicators

The general data of parturients (age, number of pregnancies, bleeding volume, labor, ethnicity, cultural level, and occupation) and newborns (gender, head circumference, blood sugar, weight, and 1 min and 5 min Apgar scores) were compared between the two groups.

The *Edinburgh Postpartum Depression Scale* [15] was adopted to evaluate and compare the postpartum depression of parturients. The total score was 30 points, and there were 10 items in total. The four options of each item were never, occasionally, often, and always, counted as 0, 1, 2, and 3 points, respectively. The first two items were scored in the opposite way, and the depression degree score was shown in Table 1.

The lactation (lactation amount and first lactation time (FLT)), breastfeeding conditions, uterine involution (days for uterine involution and descent of uterine fundus (DUF)), postpartum duration of lochia (DOL), and *Visual Analogue Scale* (VAS) score of parturients were compared and analyzed.

### 2.6. Statistical Analysis

The data was analyzed by SPSS 22.0. The mean ± standard deviation (^−^*x* ± *s*) was adopted to express the measurement data, and the percentage (%) was to express the count data. The difference was statistically significant with *P* < 0.05.

## 3. Results and Discussion

### 3.1. Comparison on General Data of Patients

The average age of parturients was 26.7 ± 5.18 years old, the average number of pregnancies was 1.77 ± 1.00, the average bleeding volume was 204.21 ± 48.38 mL, and the average delivery period was 7.62 ± 3.13. Parturients with a bachelor degree or above accounted for 39.64%, parturients working in government units accounted for 8.13%, and parturients with Han nationality accounted for 85.36%. It can be concluded from Table 2 that the differences between the two groups of parturients were not statistically significant in terms of age, number of pregnancies, bleeding volume, labor process, ethnicity, cultural level, and occupation (*P* > 0.05). It can be acquired from Table 3 that the differences between the two groups of newborns were not statistically significant in terms of gender, head circumference, blood glucose, weight, and Apgar scores at 1 min and 5 min (*P* > 0.05). The two groups were comparable.

### 3.2. Comparison on Postpartum Depression of Parturients

The occurrence of postpartum depression may cause parturients to be pessimistic and may cause parturients to have suicidal tendencies in severe case. Moreover, surveys have shown that the incidence of parturients postpartum depression in my country is about 25%, and it will relapse repeatedly in the later stage [16]. Studies have shown that fluctuations in the levels of estrogen and progesterone in parturients can easily cause emotional disturbances in parturients, and SSC can relieve the anxiety and depression of parturients. In this study, the parturients of the Exp group were subjected to SSC on the basis of routine care, and then the Edinburgh Postpartum Fepression Scale was adopted to evaluate the postpartum depression during the follow-up visit. The evaluation results were shown in Figure 1.

As illustrated in Figure 1, parturients with no or very mild, mild, moderate, and severe depression accounted for 55%, 17.86%, 25.71%, and 1.43% in the Con group, respectively, and those in the Exp group accounted for 85%, 4.29%, 10.71%, and 0%, respectively. It was found that the number of parturients with normal, mild, and moderate depression showed remarkable difference (*P* < 0.05), but the difference in severe depression was not visible (*P* > 0.05). It shows that SSC can obviously alleviate the postpartum depression of parturients. Such results are consistent with the viewpoint of Cho et al. (2021) [17], who thought that the contact during SSC and the sucking of baby can stimulate the production of hormones in the parturients, thereby stabilizing the mood of the parturients and increasing the connection between mother and baby for faster breastfeeding.

### 3.3. Comparison of Postpartum Physical Rehabilitation between the Two Groups

In order to explore the physical recovery of parturients after receiving nursing care, this article records and compares the lactation status, newborn feeding status, and uterine involution status of the parturients. The main function of the breast is to provide an important physiological organ for the offspring of mammals. During pregnancy, there is very little milk secretion, but the secretion of milk begins under the action of estrogen and progesterone after childbirth. After the cesarean section, parturients have undergone major changes both physically and psychologically, which seriously affects the secretion of milk. Studies have shown that compared with cesarean section parturients, the amount of lactation in normal parturients is more, the lactation time will be earlier, and the proportion of breastfeeding after delivery is higher [18]. In this study, the lactation amount and FLT of the two sets of parturients were compared after SSC on cesarean section parturients, and the results were shown in Figures 2 and 3.

As given in Figure 2, there were 27, 55, and 58 parturients with adequate, moderate, and insufficient lactation in the Con group, and 53, 61, and 26 parturients with adequate, moderate, and insufficient lactation in the Exp group, respectively. The comparison indicated that the number of parturients with adequate lactation in the Exp group was remarkably more (*P* < 0.05).  Figure 3 illustrated that the FLT of parturients in the Exp group (41.25 ± 4.81 h) was much shorter in contrast to the FLT in the Con group (58.43 ± 5.43 h), showing statistical difference (*P* < 0.05). It shows that SSC can promote the breast lactation in cesarean section parturients after delivery. The follow-up and record on the postpartum breastfeeding of parturients were shown in Figure 4.

As shown in Figure 4, the first BFSR (78.57%), 0.5 h starting BFR (57.14%), 1.5 h completing BFR (79.29%), predischarge BFR (74.29%), and postdischarge BFR (96.43%) of parturients in the Exp group were obviously higher, and those in the Con group were 58.57%, 35.71%, 56.43%, 45%, and 70.7%, respectively, sowing statistically visible differences (*P* < 0.05). Such results are consistent with the view of Ghojazadeh et al. (2019) [19], which pointed out that after the newborn was born, parturients continued to make SSC with the baby prematurely, which was conducive to the effective breast sucking of the baby, and can promote the production of lactation, thereby promoting breast lactation under stimulation and increasing BFR.

The process of restoring the uterus to an unpregnant state after delivery is called uterine involution. The original uterine involution takes time, and it usually takes about 1 week to recover. However, the existence of the surgical incision seriously affects the contraction of the uterus and delays the time of uterine repair due to the influence of the cesarean section on the body of the parturients. After SSC on cesarean section parturients, the days for uterine involution and the DUF of parturients were compared, and the results were given in Figures 5 and 6.

As illustrated in Figure 5, the days for uterine involution for parturients in the Exp group were shorter (6.96 ± 1.13 days vs. 9.47 ± 1.75 days), showing statistically obvious difference (*P* < 0.05).  Figure 6 reveals that the 24 h-DUF for parturients in the Exp group was obviously larger (3.17 ± 0.26 mm vs. 1.56 ± 0.43 mm) (*P* < 0.05). Such results were consistent with the viewpoint of Abultdinova et al. (2020) [20], who pointed out that performing SSC on parturients was beneficial to uterine involution due to secretion of prostaglandins under the stimulation of newborn suckling.

### 3.4. Comparison of the DOL and VAS Pain Score between the Two Groups

In addition to affecting uterine involution, cesarean section surgery can also cause uterine bleeding and inflammation and prolong the duration of lochia, which in turn affects the health of parturients [21]. Finally, in order to better observe the physical recovery of parturients, in this study, it compared the duration of postpartum lochia between the two groups of parturients after cesarean section women were given skin contact care, and the results were given in Figure 7.

Figure 7 illustrates that the postpartum DOL of parturients in the Exp group (33.21 ± 5.32 days) was much lower compared with the DOL in the Con group (25.32 ± 3.54 days), and the difference was statistically notable (*P* < 0.05). Such findings were consistent with the results of Katayama et al. (2020) [22]. When SSC is applied to parturients, the secretion of prostaglandin can alleviate chronic uterine inflammation. Later, the postpartum VAS scores of parturients were compared, and the results were shown in Figure 8.

Figure 8 suggests that the postpartum VAS score of parturients was extreme lower in the Exp group (4.88 ± 0.32 points vs. 3.41 ± 0.53 points), and the difference was statistically observable (*P* < 0.05). It shows that SSC can effectively alleviate the postpartum pain in cesarean section parturients.

## 4. Conclusion

This study is aimed at analyzing the effect of skin contact nursing on postoperative depression and physical recovery of cesarean section women. 280 pairs of parturients and newborns undergoing cesarean section were selected as the research objects, and they were randomly divided into two groups. The control group received routine care, and the experimental group received skin contact care on the basis of routine care. By comparing the two groups of parturients with postpartum depression status, lactation status, breastfeeding status, uterine involution, duration of lochia, and VAS pain score, it was found that skin contact care could significantly relieve postpartum depression in uterine parturient women, promote breast lactation, increase breastfeeding rate, facilitate uterine involution, relieve chronic uterine inflammation and postpartum pain, and have clinical application and promotion value. The shortcomings of this article are that the research sample is small, and the applicability of the results has certain limitations. The sample size can be expanded in the follow-up. All in all, this research provides a valuable clinical trial reference for the research of skin contact nursing on the body recovery and depression of cesarean section women.

## Figures and Tables

**Figure 1:** Comparison on postpartum depression of parturients.

**Figure 2:** Comparison on lactation of parturients. Note: ^∗^ suggested *P* < 0.05 in contrast to the Con group.

**Figure 3:** Comparison on breastfeeding conditions of parturients. Note: ^∗^ suggested *P* < 0.05 in contrast to the Con group.

**Figure 4:** Comparison on postpartum breastfeeding of parturients. Note: ^∗^ suggested *P* < 0.05 in contrast to the Con group.

**Figure 5:** Comparison on days for uterine involution of parturients. Note: ^∗^ suggested *P* < 0.05 in contrast to the Con group.

**Figure 6:** Comparison on DUF of parturients. Note: ^∗^ suggested *P* < 0.05 in contrast to the Con group.

**Figure 7:** Comparison on the postpartum DOL. Note: ^∗^ suggested *P* < 0.05 in contrast to the Con group.

**Figure 8:** Comparison on the postpartum VAS score. Note: ^∗^ suggested *P* < 0.05 in contrast to the Con group.

**Table 1:** Scores on degree of depression.

Degree	Score (points)
No or very mild	≤5
Mild	6 ~ 9
Moderate	10~13
Severe	≥13

**Table 2:** Comparison on general data of patients.

Item	Con group	Exp group	*t*/*χ*^2^	*P*
Age (years old)	26.67 ± 5.33	26.73 ± 5.02	0.074	0.522
Number of pregnancies (times)	1.76 ± 0.98	1.77 ± 1.02	-0.021	0.678
Bleeding volume (mL)	203.43 ± 50.32	204.98 ± 46.43	0.985	0.786
Duration of delivery (hours)	7.67 ± 3.02	7.59 ± 3.23	0.432	0.253
Nationality			0.674	0.533
Han	119	120		
Other	21	20		
Education level			1.93	0.74
High school and below	86	83		
Bachelor degree and above	54	57		
Occupation			0.643	0.921
Government units	19	20		
Self-employed entrepreneurs	43	45		
Other	78	75		

**Table 3:** Comparison on general data of newborns.

Item	Con group	Exp group	*t*/*χ*^2^	*P*
Gender			0.182	0.543
Males	65	68		
Females	75	72		
Weight (g)	3385.3 ± 335.3	3335.4 ± 374.8	0.878	1.211
Head circumference (cm)	34.3 ± 0.48	34.2 ± 0.33	1.322	0.628
Blood glucose (mmol/L)	4.68 ± 1.21	4.70 ± 0.97	0.789	0.242
1 min Apgar score	8.89 ± 0.21	8.92 ± 0.13	-0.434	0.253
5 min Apgar score	9.94 ± 0.15	9.95 ± 0.24	-0.364	0.097

## Data Availability

The data underlying the results presented in the study are available within the manuscript.
